This article has been retracted.

# The Use of Hellinger Distance Undersampling Model to Improve the Classification of Disease Class in Imbalanced Medical Datasets

**DOI:** 10.1155/2020/8824625

**Published:** 2020-11-04

**Authors:** Zina Z. R. Al-Shamaa, Sefer Kurnaz, Adil Deniz Duru, Nadia Peppa, Alex H. Mirnezami, Zaed Z. R. Hamady

**Affiliations:** ^1^Graduate School of Science and Engineering, Altınbaş University, Istanbul, Turkey; ^2^Sports and Health Sciences Department, Marmara University, Istanbul, Turkey; ^3^Southampton University Hospital NHSFT, Southampton, UK

## Abstract

Imbalanced class distribution in the medical dataset is a challenging task that hinders classifying disease correctly. It emerges when the number of healthy class instances being much larger than the disease class instances. To solve this problem, we proposed undersampling the healthy class instances to improve disease class classification. This model is named Hellinger Distance Undersampling (HDUS). It employs the Hellinger Distance to measure the resemblance between majority class instance and its neighbouring minority class instances to separate classes effectively and boost the discrimination power for each class. An extensive experiment has been conducted on four imbalanced medical datasets using three classifiers to compare HDUS with a baseline model and three state-of-the-art undersampling models. The outcomes display that HDUS can perform better than other models in terms of sensitivity, F1 measure, and balanced accuracy.

## 1. Introduction

Classification is a standard data mining process. It consists of two steps, building a model and testing a model. A classification model is built to learn from training data which is then tested to predict the category of unknown samples. Most classification algorithms were mainly built to classify the balanced dataset, whereas a problem occurs when a dataset is imbalanced, which degrades the recognition power of the classifier [1]. The imbalanced problem appears when the data is composed of very different sample numbers for the various classes; i.e., the number of samples of one class is greater than those in the second class, the former is called the majority class, and the latter is called the minority class [2]. Imbalanced datasets usually influence the classification process. If the problems of imbalanced class distribution are not addressed before implementing the classification procedures, the classifier appears to be biased towards the majority class cases while ignoring to classify the minority class cases correctly [3]. However, the problems of classifying imbalanced data often occur in real-life applications such as analyzing medical datasets, where the cases of patients with the disease are significantly lower than those without the disease. For instance, in cancer detection, the cases of patients diagnosed with cancer are much smaller than those of patients who do not have cancer [4]. The classification model to predict cancer results in lower classification performance of abnormal class and incorrect prediction disease which leads to serious health risk.

In general, the problem of classifying imbalanced data is due to the lack of training with a few minority class samples which are inadequate to predict accurately [5]. Previous studies have proposed resampling techniques to solve the problem of class imbalance. These techniques are mainly categorized into oversampling and undersampling [6]. The oversampling method is aimed at generating samples for the minority class [7], and the undersampling method is aimed at reducing samples for the majority class [8].

In this work, we propose a novel undersampling technique, named the Hellinger Distance Undersampling (HDUS) model, aimed at solving the imbalanced classification problem in medical datasets. The proposed model reduces healthy class samples to improve the classifying performance of the rare disease class. It adopts the Hellinger distance to measure the similarity between majority class instance and its neighbouring minority class instances, then chooses a number of the highest Hellinger distance values, and sums them up to be a similarity value for each majority instance. Finally, the model selects a subset from the majority instances, having top similarity values, and combined with the original minority class instances. This model could effectively separate major class instances and minor class instances and boost the discrimination power for each class, thereby improving the classification accuracy for rare class. We compared the HDUS with four models, including a baseline model without using any sampling technique and three state-of-the-art undersampling models. The experiment was conducted on four imbalanced medical datasets using three classifiers.

The remainder of this paper is organized as follows.  Section 2 mentions a related work.  Section 3 presents the proposed model.  Section 4 reviews the experiment setup.  Section 5 presents the results of the experiment.  Section 6 demonstrates the discussion of the results.  Section 7 is the conclusion of the study.

## 2. Related Work

Recently, the problem of imbalanced classification has drawn much attention in the literature because the traditional classification algorithms were not initially built to train the imbalanced dataset [9]. This problem usually emerges from the different distribution of classes in the feature space. Furthermore, there are some other problematic features of imbalanced datasets such as overlapping samples, small disjoints, and small sample sizes. The overlapping denotes to the data samples in various classes that overlap in the feature space. The small disjoint denotes to the few samples in the minority class that are spread separately in the feature space. Finally, the small sample sizes refer to an insufficient number of data samples in the minority class. The aforementioned imbalanced features would raise the complexity of the classifier, which in turn makes it difficult to classify the minority class samples correctly [5, 10].

To overcome the imbalanced data problem, current approaches may be categorized to the algorithm level and data level. The first group works to change the classification algorithm, to support the minority class cases, by specifying weights to cases from various classes or by ensemble methods [11, 12]. The second group applies before the classification procedure to modify the distribution of imbalanced dataset through data sampling techniques [13].

Previous studies indicated that solving the imbalanced problem at the data level is simple and efficient for unbalanced classification [1]. Therefore, data sampling techniques have been widely used to alleviate the unbalanced classification problem by modifying the distribution of classes in the training dataset. Generally, sampling techniques are categorized into over- and undersampling [14]. The oversampling technique is aimed at generating instances artificially for a minority class by adding copies of already existing data from minor class instances [7]. Many methods of oversampling have been applied earlier. Random oversampling (ROS) is a common oversample approach that randomly adds samples to the minor class. Although ROS adjusts the class distribution, it may increase the overfitting problem by making similar copies of the minor class that influence the classification process [14]. Another standard oversample approach is the synthetic minority oversampling technique (SMOTE) [15]. It is used to generate artificial samples. Unlike ROS, SMOTE avoids the overfitting problem, but it may cause the overlapping with the surrounding samples that increase the overall training data size and hinder the training process [16, 17]. Generally, with the oversampling technique, the problem of an imbalanced class is diluted, but the training data is going to get more crowded. Therefore, the classification performance is affected [18].

Undersampling is another reasonable data sampling technique which attempts to reduce the number of samples in the majority class. The undersampling concept is how to eliminate majority class instances in a manner that retains the practical distinction among classes [8]. Numerous undersampling methods have been implemented and used earlier. The most naive approach is random undersampling (RUS), which eliminates instances from major class randomly. It tends to balance the distribution of classes but causes waste of valuable information that could be essential for the classification process [14]. Tomek link (Tml) is another undersampling method used to address the overlapping problem. It looks for pairs of samples belonging to different classes but are each other's nearest neighbour and eliminates the majority sample of the pair [19]. Another method is the edited nearest neighbour, which is applied to eliminate major class samples based on the nearest *K* neighbour that belongs to the minor samples. When the number of neighbours in each major class is higher in the minor class, the major class sample shall be omitted as noise or borderline [20].

Previous research studies revealed that there is no optimal rule to attain the best fit with over- or undersampling. They have shown that usually undersampling process of the major class is used to outperform the results obtained through the oversampling of the minor class [15]. More than that, as the data size has been increasing, the undersampling method would be a better option than the oversampling method [21]. Instance selection was used in previous studies to remove the outlier from the training dataset, which can make the classifier perform better than the original dataset [22–24]. However, the existing instance selection techniques have programmed to choose a portion of the initial dataset which cannot be used directly to choose instances from just one class of the dataset, such as selecting from the major class instances. Kubat and Matwin in [25] proposed one-sided instance selection to remove noise samples, redundant samples, and borderline samples from the majority class while keeping the original samples belonging to the minority class.

Recently, a lot of undersampling methods have been reported in the literature to improve the imbalanced data classification. Tsai et al. in [10] introduced an undersampling method by clustering the majority class into groups of similar data samples; then, the instance selection extracts the nonrepresentative data samples from each group. Nwe and Lynn in [20] suggested an undersampling approach began by determining the closest major class neighbours to each minor class sample, then evaluating the number of correlation of each neighbour from the major class with the minor class samples. Finally, the required number of major class instances is taken from the number of correlations. Besides, the authors in [26] adopted the one-sided undersampling technique. They proposed a method for reducing the major class size that modifies the distribution of initial imbalanced classes by measuring the similarities of each major class case with the corresponding minor class cases. The method effectively separates the major and minor class cases to optimize the identity value for each class.

## 3. Proposed Model

The work is aimed at providing a method that handles the problem of imbalanced data distribution which affects classification performance of minority class samples. In the imbalanced dataset, the class with a larger number of instances takes up most of the space. Unequal class distribution makes the classifier to be inadequately qualified to classify the smaller class instances, and the class with a larger number of instances overlaps the identification ability of the class with a smaller number of instances. In this case, the classifier would favour the majority class instances and scoring false high accuracy.

In this work, we proposed an undersampling model by following the principle of one-sided selection to extract instances from the major class, while the data in the minor class will remain without change. This is based on the premise that it is better to keep the instances of a minor class as real as they are, in such a manner that no greater or no less quantity is exercised on them. So, the classifier will be provided by an accurate recognition power for the original minor class samples.

Instance selection in the undersampling technique depends on how to select majority class instances in a manner that retains the compatible distinction among classes. In our proposed model, we used Hellinger distance (HD) [27, 28] to choose instances from the major class based on their Hellinger similarity degree with the minor class instances. Hellinger distance is a measure of the variance in distribution [29]. In [30], Cieslak et al. demonstrated analytically that HD is very robust in the presence of a skew distribution of class and it is not affected by the class imbalanced rate due to its isometric contours. This is the motivation of using HD in our proposed method. To express the equation of Hellinger distance, let *a*(*x*) and *b*(*x*) be two probability functions; then the HD between *a*(*x*) and *b*(*x*) can be expressed as follows:

(1) $$\begin{array}{c} \text{HD}\left(a,b\right)=\frac{1}{\sqrt{2\;}}\sqrt{\int {\left(\sqrt{a\left(x\right)}-\sqrt{b\left(x\right)}\right)}^{2}dx}. \end{array}$$

Considering the problem of classification of the imbalanced class dataset and being motivated by the properties of the HD, we proposed an undersampling model using Hellinger similarity measure. The proposed model works to reduce the number of major class instances, aimed at upgrading the prediction performance of minority class which is the class of teh highest interest in medical datasets.  Algorithm 1 the pseudocode of the proposed HDUS model:

## 4. Experiment Setup

In this section, we display the details of the experiment to test the proposed HDUS model. We present the nature of the datasets, the used classification algorithms, the evaluation metrics, and the undersampling methods used for comparison.

The code for the whole experiment was conducted in Python Programming language and spyder tools using the available utilities to provide all the necessary preprocessing and classification techniques besides the evaluation functions.

### 4.1. Datasets

In this work, we have exercised four imbalanced medical datasets to evaluate the performance of the suggested (HDUS) model. For each dataset, the number of features (attributes), the number of instances, the number of majority cases, and the number of minority cases are presented. These datasets are described in the following.

#### 4.1.1. A Novel Colorectal Cancer Dataset (CRC)

This dataset is from the Southampton University Hospital and has been used with approval from the responsible surgeon (co-author), and the data are all anonymous. The data are for patients having primary cancer at 12 colorectal sites, who then have cancer resection surgery. There are 1005 instances (patients), each of which acts as a record of a single patient with 14 features (attributes), including the target label. Out of 1005 instances, 760 are for patients having primary CRC who do not have metastasis, representing the majority samples, and another 245 cases are for patients having primary CRC growing to metastasis in other organs of the body, representing the minority samples. The data type is categorical (groups into multiple categories) and mapped to numeric values.  Table 1 shows the features of colorectal cancer dataset.

#### 4.1.2. PIMA Indians Dataset

The dataset of PIMA Indians was taken from the UCI machine learning repository [31]. It has nine features, including the class feature. The class feature indicates if there are patients with diabetes or not. The dataset has 768 samples, including 268 having diabetes (the minority samples) and 500 without diabetes (the majority samples). The information of features is shown in Table 2.

#### 4.1.3. Thoracic Surgery Dataset (THS)

The thoracic data was taken from the UCI machine learning repository [31]. This data was collected from patients who experienced tumour resections for primary lung cancer. The dataset has 17 features, including the class feature. It has 470 samples, including 70 patients who died during the one year after surgery (the minority samples) and 400 who are alive (the majority samples). The information of features is shown in Table 3.

#### 4.1.4. Breast Cancer (BC) Dataset

The BC dataset was taken from the UCI machine learning repository [31] which is provided by the Oncology Institute. It has ten features, including the class feature. The dataset indicates if a breast cancer recurred or not. The dataset has 286 samples, including 85 cases of the minority class and 201 cases of the majority class. The information of features is shown in Table 4.

### 4.2. Classification Data Mining Algorithms

In this study, three classification algorithms with different characteristics were explored: decision tree (DT), Support Vector Machine (SVM), and *K*-Nearest Neighbour (KNN). The primary purpose of using these classifiers was to evaluate the performance of the proposed model on four imbalanced medical datasets. The experiment was initially done on a CRC dataset and then tested on three datasets selected from the UCI repository.

#### 4.2.1. *K*-Nearest Neighbour (KNN)

KNN is a classification technique that relies on feature similarity measures to find the closest neighbours. For the classification of a new point, the KNN reviews each training sample as a tuple (*X*) with the particular label denoting its class. KNN counts the spaces between *X* and all training tuples, then specifies to *X* the maximum repeat class in the nearest *k* tuple [32].

#### 4.2.2. Support Vector Machine (SVM)

SVM is a supervised kernel-based classification algorithm that can be used for binary classification problems. It uses a mathematical function to define an optimal hyperplane that splits two classes in a training dataset with a maximum margin. Then, SVM increases the space between the closest training data points (support vectors) and the class boundaries trying to find the optimal hyperplane that removes some insignificant data from the training data set. However, when the data is intrinsically nonlinear, SVM will use kernel function to construct a separating hyperplane that transforms the data from the original dimension into a high-dimensional space. Popularly used kernel functions are the linear, polynomial, sigmoid, and Gaussian kernel [33, 34].

#### 4.2.3. Decision Tree (DT)

A decision tree classifier involves several simpler decisions to build a tree model. The tree model builds three types of nodes: root, internal, and leaf. The root represents the starting point which has no incoming edges but outgoing edges. The internal nodes are represented by the data attribute, which has only one incoming branch and at least two leaving branches for each possible attribute. The leaf nodes are represented by the classes. These patterns of the decision tree express sets of if-then rules that can be employed to classify novel samples [35].

### 4.3. Evaluation Metrics

A classifier is, typically, evaluated by a confusion matrix which contains four values from classification outputs that report the number of True Positive (TP), True Negative (TN), False Positive (FP), and False Negative (FN). The TP refers to the rate of correctly recognizing the rare positive. The TN refers to the rate of correctly recognized negative. The FP refers to the rate of frequent negative incorrectly recognized as rare positive, and the FN refers to the rate of rare positive incorrectly recognized as frequent negative. In the experiment, the minority class refers to positive and the majority class refers to negative. The most used performance measure of classification tasks is accuracy. However, it is not an appropriate metric when evaluating the imbalanced class distributions because the classifier has a strong bias towards the majority class and fails to classify the few samples of minority class [36].

More proper metrics could be used to assess the performance measurement of classifying imbalanced class distribution, such as sensitivity or recall (True positive rate (TPR)), specificity (True negative rate (TNR)) [37], precision (positive predictive value (PPV)) [32], F1-measure [35], and balanced accuracy (BACC) [38].

These metrics are given by equations in (2) as follows:

(2) $$\begin{array}{c} \text{TPR}=\frac{\text{TP}}{\text{TP}+\text{FN}},\\ \text{TNR}=\frac{\text{TN}}{\text{TN}+\text{FP}},\\ \text{PPV}=\frac{\text{TP}}{\text{TP}+\text{FP}},\\ \text{F}1\text{\_m}=\frac{\;2\times \text{TPR}\times \text{PPV }}{\text{TPR}+\text{PPV}},\\ \text{BACC}=\frac{\text{TPR}+\text{TNR}}{2}. \end{array}$$

To ensure an unbiased evaluation of the models, the *n*-fold cross-validation is used as an evaluation criterion. In *n*-fold cross-validation, the data were divided into *n* equal folds, then the model was trained on all folds except one fold as a validation set on which the prepared model was tested. The process repeats so that each fold gets an opportunity to act as the test set. Then, the *n*-test outcome was averaged [35]. In our work, the *n* value is set to 5.

### 4.4. Comparative Method

To allow a fear valuation of the validity of our proposed method, HDUS is compared against three other undersampling methods:

- Tomek link (Tml): it is aimed at removing the noise and border points from majority class instances by examining pairs of samples belonging to different classes but are each other's nearest neighbour and eliminates the majority sample of the pair [19].
- Random undersampling (RUS): it eliminates instances from major class randomly until the desired balance of class distribution is achieved [14].
- Edited nearest neighbour (ENN): the basic idea of ENN is to eliminate samples of the major class based on the *K*-Nearest Neighbour that belong to the minor samples. If the number of neighbours is predominant in each majority instance from minority instances, certain instances of the majority class are eliminated as overlap instances [20].

## 5. Results Analysis

To investigate the performance measures of the proposed HDUS method, we used four imbalanced medical datasets using three classification algorithms including DT, SVM, and KNN and they were compared with the baseline model (without any resampling method) and with three state-of-the-art undersampling methods (Tomek link, RUS, and ENN). The results of the four datasets (CRC, PIMA, THS, and BC) are shown in Tables 5–8, respectively, in terms of sensitivity, specificity, precision, F1 measure, and balanced accuracy.

As shown in Tables 5–8, the first column of the baseline model confirms that the imbalanced classification problem exists in all used datasets. This presents a low average rate of sensitivity to predict minority class; it ranges from 7.94% in the THS dataset to 39.7% in the PIMA dataset, while it assigns a high average rate of specificity to predict the instances of the majority class.

The 2^nd^, 3^rd^, and 4^th^ columns of the tables represent the result of used undersampling methods: Tomek link, RUS and ENN, respectively. We can observe the improvement achieved by using these methods, as expressed by the values of sensitivity that reflects the ability of the models to detect the class of interest, i.e., the minor class. Although the Tomek link obtained worse performance in all datasets, it is better than the baseline model except in the THS dataset, which scored lower than the baseline model.

More improvement is achieved in the 5^th^ column of all tables by the proposed HDUS method in terms of sensitivity, F1_m, and Bacc. It can be observed that the HDUS performance shows significant improvement over the baseline and the three undersampling methods. The HDUS results in the top rate of sensitivity overall datasets (that refers to the highest ability to detect the class of interest, i.e., the minority class). It scores over 80% in both CRC and PIMA, near 70% in BC and near 60% in THS which is the lowest sensitivity. It also results in the highest rate for both F1_m and balanced accuracy.

## 6. Discussion

This study discussed about a preprocessing undersampling method named HDUS. The model handles the class inequality problem in medical datasets to improve the prediction performance of the minority class samples by using the instance selection based Hellinger distance similarity measure.

It is crucial to refer to the need for handling the issue of class inequality by choosing appropriate approaches that address the skewed distributions of data. As noted in the previous section, the baseline classification of original datasets shows a very high value of specificity to predict the majority class samples but a very poor sensitivity to predict the minority class samples, which is the class of interest in the imbalanced medical datasets. The use of traditional undersampling techniques shows good progress, mainly by RUS. However, using RUS seems to be not convenient since it eliminates meaningful samples randomly and can also cause overfitting due to the expanding of scar samples without limitations [26]. The performance of ENN is lower than that of RUS except in PIMA dataset, and Tml is the worst one in the experiment. However, the proposed HDUS method has proved to overcome all the other methods in the experiment for all datasets due to the robust measure of Hellinger distance which has the property of skew intensive that is not affected by the class imbalance [30].

To simplify the comparison among the different undersampling methods used in the experiment and to evaluate their efficiency, Figures 1–3 provide a graphical representation for the average values of (sensitivity, F1_m, and Bacc) resulting from the five models applied on four imbalanced medical datasets. As can be seen from the figures, the performances vary when different undersampling techniques are utilized. From Figure 1, it is evident that our HDUS method has made good progress in predicting minority class samples on all datasets in terms of sensitivity. The similar situation can be found through Figure 2 for F1_m, which is the trade-off between precision and recall, and Figure 3 for Bacc, which is the trade-off between sensitivity and specificity.

Regarding the classification methods, it is worth to remark that the benefit of carrying out classification increases when the class imbalance issue is appropriately addressed. In our experiment, different classification algorithms may benefit from the adoption of the HDUS model. In particular, DT achieves the best performance with HDUS. It also obtained the best results with Tml and ENN, whereas SVM is more appropriate for the RUS method. As shown in Table 9, the average results of used classifiers with experimented undersampling methods in the four datasets achieved improvement in predicting the minority class samples through sensitivity, F1_m, and Bacc.

Finally, the results of the proposed HDUS model should be considered as a preliminary experiment, but a promising method in the application of undersampling the imbalanced medical dataset to improve the classification performance of minor class samples.

## 7. Conclusion

This paper proposed a novel model, HDUS, that handles the imbalanced classification problem in the medical datasets to improve the classification of the minority disease class. HDUS works to reduce the majority class instances by using the Hellinger distance to calculate the similarity between majority class instance and minority class instances. Then, HDUS selects a subset from the majority class instances having the highest similarity values that are shown to perform well in combination with the original minority class instances. The experiment was conducted on four imbalanced medical datasets using three classifiers to compare HDUS with a baseline model and three selective undersampling models. The performance results show that HDUS could achieve significant improvement over the selective models in terms of sensitivity, which is highly desirable in the medical domain, F1_measure, and balanced accuracy. HDUS has proved to be a promising model for rebalancing the imbalanced medical datasets which contain a few but important cases of disease class.

In a future work, we encourage comparing HDUS with other sampling techniques for the same classifiers or using other classifiers or even utilizing a larger number of medical datasets with different characteristics. We also suggest integrating the proposed model with other sampling techniques to handle the imbalanced classification problem in medical datasets.

## Figures and Tables

**Figure 1:** The average sensitivity results using models (baseline, Tml, RUS, ENN, and HDUS) for four datasets.

**Figure 2:** The average F1_m results using models (baseline, Tml, RUS, ENN, and HDUS) for four datasets.

**Figure 3:** The average Bacc results using models (baseline, Tml, RUS, ENN, and HDUS) for four datasets.

**Algorithm 1:** Algorithm 1: Hellinger Distance Undersampling (HDUS) pseudocode

**Table 1:** The features of colorectal cancer dataset.

No.	Attribute name	Data type
1	Tumour site (in colorectal)	Categorical
2	Surgery type	Categorical
3	Operation type (on which part of colorectal the operation was done)	Categorical
4	Differentiation	Categorical
5	Dukes stage of tumour	Categorical
6	T stage 5th edition	Categorical
7	N stage 5th edition	Categorical
8	EMVI	Categorical
9	Tumour perforation	Categorical
10	Resection margin	Categorical
11	Neoadjuvant therapy n-CRT	Categorical
12	Chemotherapy	Categorical
13	Radiotherapy	Categorical
14	CRC metastasis (class)	Categorical

**Table 2:** The features of PIMA Indian dataset.

No.	Attribute name	Data type
1	Number of times pregnant	Numeric
2	Plasma glucose concentration	Numeric
3	Diastolic blood pressure	Numeric
4	Triceps skinfold thickness	Numeric
5	Amount of insulin	Numeric
6	Body mass index	Numeric
7	Diabetes pedigree function	Numeric
8	Age	Numeric
9	Class	Categorical

**Table 3:** The features of THS dataset.

No.	Attribute name	Data type
1	Diagnosis	Categorical
2	Forced vital capacity	Numeric
3	A volume that has been exhaled at the end of the first of forced expiration	Numeric
4	Performance status	Categorical
5	Pain before surgery	Categorical
6	Hemoptysis before surgery	Categorical
7	Dyspnoea before surgery	Categorical
8	Cough before surgery	Categorical
9	Weakness before surgery	Categorical
10	Size of the original tumour	Categorical
11	Type 2 diabetes mellitus	Categorical
12	Myocardial infarction up to six months	Categorical
13	Peripheral arterial diseases	Categorical
14	Smoking	Categorical
15	Asthma	Categorical
16	Age at surgery	Numeric
17	One-year survival period (class)	Categorical

**Table 4:** The features of BC dataset.

No.	Attribute name	Data type
1	Tumor size	Categorical
2	Inv nodes	Categorical
3	Node caps	Categorical
4	Menopause	Categorical
5	deg malig	Categorical
6	Breast side	Categorical
7	Breast quad	Categorical
8	Irradiat	Categorical
9	Age	Categorical
10	Class (recurrence/no-recurrence)	Categorical

**Table 5:** Evaluation results for CRC dataset using classifiers (KNN, SVM, and DT) and models (baseline, Tml, RUS, ENN, and HDUS).

CRC		Baseline	Tml	RUS	ENN	HDUS
KNN	Sensitivity (%)	29.41	37.25	62.75	62.75	80.35
	Specificity (%)	85.38	75.38	60	60.31	50.23
	Precision (%)	44.12	37.25	38.1	38.51	33.91
	F1_m (%)	35.29	37.25	47.41	47.73	47.69
	Bacc (%)	57.4	56.32	61.38	61.53	65.29

SVM	Sensitivity (%)	5.88	29.41	62.75	47.06	76.40
	Specificity (%)	92.31	82.31	54.62	70.77	55.85
	Precision (%)	23.08	39.47	35.16	38.71	35.40
	F1_m (%)	9.37	33.71	45.07	42.48	48.38
	Bacc (%)	49.1	55.86	58.68	58.91	66.13

DT	Sensitivity (%)	35.29	45.1	62.75	66.67	81.00
	Specificity (%)	68.46	59.23	46.92	43.85	56.91
	Precision (%)	30.51	30.26	31.68	31.78	39.90
	F1_m (%)	32.73	36.22	42.1	43.04	53.46
	Bacc (%)	51.88	52.16	54.83	55.26	68.96

AVG	Sensitivity (%)	23.53	37.25	62.75	58.83	79.25
	Specificity (%)	82.05	72.31	53.85	58.31	54.33
	Precision (%)	32.57	35.66	34.98	36.33	36.40
	F1_m (%)	27.32	36.44	44.92	44.92	49.85
	Bacc (%)	52.79	54.78	58.3	58.57	66.79

**Table 6:** Evaluation results for PIMA dataset using classifiers (KNN, SVM, and DT) and models (baseline, Tml, RUS, ENN, and HDUS).

PIMA		Baseline	Tml	RUS	ENN	HDUS
KNN	Sensitivity (%)	60.06	64.52	70.77	70.57	83.87
	Specificity (%)	83.85	80	73.85	74.92	62.50
	Precision (%)	63.16	56.61	56.41	56.46	50.35
	F1_m (%)	61.57	60.31	62.78	62.73	62.92
	Bacc (%)	70.96	72.26	72.41	72.75	73.19

SVM	Sensitivity (%)	0	66.13	74.42	74	79.03
	Specificity (%)	100	83.85	73.85	76.92	71.50
	Precision (%)	0	58.13	58.54	58.04	57.00
	F1_m (%)	0	61.87	65.53	65.06	66.23
	Bacc (%)	50	74.99	74.63	75.86	75.27

DT	Sensitivity (%)	61.29	69.35	70.97	70.97	91.90
	Specificity (%)	79.23	66.92	58.46	68.46	66.77
	Precision (%)	58.46	50	44.9	50.76	56.98
	F1_m (%)	59.84	58.11	55	59.19	70.34
	Bacc (%)	70.26	68.14	64.71	69.71	79.34

AVG	Sensitivity (%)	39.78	66.67	72.05	71.85	84.93
	Specificity (%)	87.69	76.92	68.72	73.43	66.92
	Precision (%)	40.54	54.91	53.28	54.09	54.78
	F1_m (%)	40.16	60.22	61.26	61.72	66.50
	Bacc (%)	63.74	71.8	70.58	72.77	75.93

**Table 7:** Evaluation results for THS dataset using classifiers (KNN, SVM, and DT) and models (baseline, Tml, RUS, ENN, and HDUS).

THS		Baseline	Tml	RUS	ENN	HDUS
KNN	Sensitivity (%)	0.00	0.00	42.86	4.76	23.81
	Specificity (%)	100.00	98.97	60.82	91.75	75.26
	Precision (%)	0.00	0.00	19.15	11.11	19.24
	F1_m (%)	0.00	0.00	26.47	6.67	21.28
	Bacc (%)	50.00	49.48	51.84	48.26	49.53

SVM	Sensitivity (%)	0.00	0.00	66.67	4.76	71.43
	Specificity (%)	100.00	100.00	47.42	91.75	44.27
	Precision (%)	0.00	0.00	21.54	11.11	21.13
	F1_m (%)	0.00	0.00	32.56	6.67	32.61
	Bacc (%)	50.00	50.00	57.04	48.26	57.84

DT	Sensitivity (%)	23.81	14.29	42.86	38.10	80.95
	Specificity (%)	87.63	91.75	48.45	81.44	40.02
	Precision (%)	29.41	27.27	15.25	30.77	25.99
	F1_m (%)	26.32	18.75	22.50	34.04	39.33
	Bacc (%)	55.72	53.02	45.66	59.77	60.48

AVG	Sensitivity (%)	7.94	4.76	50.79	15.87	58.73
	Specificity (%)	95.88	96.91	52.23	88.32	53.18
	Precision (%)	9.80	9.09	18.65	17.66	22.12
	F1_m (%)	8.77	6.25	27.18	15.79	31.07
	Bacc (%)	51.91	50.83	51.51	52.09	55.95

**Table 8:** Evaluation results for BC dataset using classifiers (KNN, SVM, and DT) and models (baseline, Tml, RUS, ENN, and HDUS).

BC		Baseline	Tml	RUS	ENN	HDUS
KNN	Sensitivity (%)	33.33	44.44	57.11	50	61.11
	Specificity (%)	84.91	70.36	65.81	70.36	73.58
	Precision (%)	42.86	40	40.74	42.86	44.00
	F1_m (%)	37.5	42.1	47.56	46.16	51.16
	Bacc (%)	59.12	57.4	61.46	60.18	67.35

SVM	Sensitivity (%)	22.22	38.89	66.67	44.44	66.67
	Specificity (%)	94.34	88.68	64.15	83.02	69.81
	Precision (%)	57.14	53.85	38.71	47.06	42.86
	F1_m (%)	32	45.16	48.98	45.71	52.17
	Bacc (%)	58.28	63.78	65.41	63.73	68.24

DT	Sensitivity (%)	38.89	38.89	44.44	44.44	77.78
	Specificity (%)	66.04	64.15	62.26	69.81	66.04
	Precision (%)	28	26.92	28.57	33.33	43.75
	F1_m (%)	32.56	31.82	34.78	38.09	56.00
	Bacc (%)	52.46	51.52	53.35	57.13	71.91

AVG	Sensitivity (%)	31.48	40.74	56.07	46.29	68.52
	Specificity (%)	81.76	74.4	64.07	74.4	69.81
	Precision (%)	42.67	40.26	36.01	41.08	43.54
	F1_m (%)	36.23	40.5	43.85	43.53	53.11
	Bacc (%)	56.62	57.57	60.07	60.35	69.17

**Table 9:** The average results using classifiers (KNN, SVM, and DT) with models (baseline, Tml, RUS, ENN, and HDUS) on four datasets.

		Baseline	Tml	RUS	ENN	HDUS
KNN	Sensitivity (%)	30.70	36.55	58.37	47.02	62.28
	Specificity (%)	88.54	81.18	65.12	74.34	65.39
	Precision (%)	37.54	33.47	38.60	37.24	36.88
	F1_m (%)	33.59	34.92	46.06	40.82	45.76
	Bacc (%)	59.37	58.87	61.77	60.68	63.84

SVM	Sensitivity (%)	7.03	33.61	67.63	42.57	73.38
	Specificity (%)	96.66	88.71	60.01	80.62	60.36
	Precision (%)	20.06	37.86	38.49	38.73	39.10
	F1_m (%)	10.34	35.19	48.03	39.98	49.85
	Bacc (%)	51.85	61.16	63.94	61.69	66.87

DT	Sensitivity (%)	39.82	41.91	55.25	55.04	82.91
	Specificity (%)	75.34	70.51	54.02	65.89	57.44
	Precision (%)	36.60	33.61	30.10	36.66	41.65
	F1_m (%)	37.86	36.23	38.60	43.59	54.79
	Bacc (%)	57.58	56.21	54.64	60.47	70.17

## Data Availability

The Colorectal Cancer Dataset is not publicly available; it is from the Southampton University Hospital and has been used with approval from the responsible surgeon (co-author), and the data are all anonymous. The datasets “PIMA”, “Thoracic surgery”, and “Breast Cancer” are openly available at the UCI Machine Learning Repository at https://archive.ics.uci.edu/ml.
